The article "The Heart of Silk Road “Xinjiang,” Its Genetic Portray, and Forensic Parameters Inferred From Autosomal STRs" was retracted in 2024. Reasons: lack of ethics approval or compliance; concerns about the welfare of human subjects.

# The Heart of Silk Road “Xinjiang,” Its Genetic Portray, and Forensic Parameters Inferred From Autosomal STRs

**DOI:** 10.3389/fgene.2021.760760

**Published:** 2021-12-17

**Authors:** Atif Adnan, Adeel Anwar, Halimureti Simayijiang, Noor Farrukh, Sibte Hadi, Chuan-Chao Wang, Jin-Feng Xuan

**Affiliations:** ^1^ Department of Forensic Genetics, School of Forensic Medicine, China Medical University, Shenyang, China; ^2^ Department of Forensic Sciences, College of Criminal Justice, Naif Arab University of Security Sciences, Riyadh, Kingdom of Saudi Arabia; ^3^ Department of Anthropology and Ethnology, School of Sociology and Anthropology, Institute of Anthropology, Xiamen University, Xiamen, China; ^4^ Department of Orthopedic Surgery, The 3rd Affiliated Hospital of Chongqing Medical University, Chongqing, China; ^5^ Department of Forensic Medicine, School of Basic Medical Sciences, Binzhou Medical University, Yantai, China; ^6^ State Key Laboratory of Cellular Stress Biology, School of Life Sciences, National Institute for Data Science in Health and Medicine, Xiamen University, Xiamen, China; ^7^ State Key Laboratory of Marine Environmental Science, Xiamen University, Xiamen, China

**Keywords:** Uyghur, Kazakh, hui, han, autosomal STRs, phylogenetics, allelic frequency database

## Abstract

The Xinjiang Uyghur Autonomous Region of China (XUARC) harbors almost 50 ethnic groups including the Uyghur (UGR: 45.84%), Han (HAN: 40.48%), Kazakh (KZK: 6.50%), Hui (HUI: 4.51%), Kyrgyz (KGZ: 0.86%), Mongol (MGL: 0.81%), Manchu (MCH: 0.11%), and Uzbek (UZK: 0.066%), which make it one of the most colorful regions with abundant cultural and genetic diversities. In our previous study, we established allelic frequency databases for 14 autosomal short tandem repeats (STRs) for four minority populations from XUARC (MCH, KGZ, MGL, and UZK) using the AmpFlSTR® Identifiler PCR Amplification Kit. In this study, we genotyped 2,121 samples using the GoldenEye™ 20A Kit (Beijing PeopleSpot Inc., Beijing, China) amplifying 19 autosomal STR loci for four major ethnic groups (UGR, HAN, KZK, and HUI). These groups make up 97.33% of the total XUARC population. The total number of alleles for all the 19 STRs in these populations ranged from 232 (HAN) to 224 (KZK). We did not observe any departures from the Hardy–Weinberg equilibrium (HWE) in these populations after sequential Bonferroni correction. We did find minimal departure from linkage equilibrium (LE) for a small number of pairwise combinations of loci. The match probabilities for the different populations ranged from 1 in 1.66 × 10^23^ (HAN) to 6.05 × 10^24^ (HUI), the combined power of exclusion ranged from 0.999 999 988 (HUI) to 0.999 999 993 (UGR), and the combined power of discrimination ranged from 0.999 999 999 999 999 999 999 983 (HAN) to 0.999 999 999 999 999 999 999 997 (UGR). Genetic distances, principal component analysis (PCA), STRUCTURE analysis, and the phylogenetic tree showed that genetic affinity among studied populations is consistent with linguistic, ethnic, and geographical classifications.

The article "The Heart of Silk Road “Xinjiang,” Its Genetic Portray, and Forensic Parameters Inferred From Autosomal STRs" was retracted in 2024. Reasons: lack of ethics approval or compliance; concerns about the welfare of human subjects.

## 1 Introduction

The Altai is a mountain range in Central and East Asia and stretches around Kazakhstan and Russia in the west while Xinjiang in the northwest China and Mongolia in the East. In ancient times, Europeans were settled on the western side and Asians on the eastern side of these mountains (Li et al., 2019). Later on, the region was used as a corridor by European and Asian populations. This corridor played an important role in the formation of new ethnic groups and diversity of populations today (Ovodov et al., 2011). The Xinjiang Uyghur Autonomous Region (XUAR) is the most diversified region in China, and it is the home of almost 50 ethnic groups. XUAR has played a vital role in the early ages because it was connecting not only the Altai mountain range corridor but also western Eurasia and eastern Eurasia (Esposito, 1999). It was also the main hub for the famous Silk Road, which linked trade between the Middle East, East Asia, Central Asia, South Asia, and Europe (Esposito, 1999). XUAR is divided into two basins, Dzungarian (North Basin) and Tarim (South Basin). Many ethnic groups, including the Uyghur (UGR), Kazakh (KZK), Hui (HUI), Han (HAN), Manchu (MCH), Mongols (MGL), Kirgiz (KGZ), and Uzbek (UZK) have lived there for hundreds of years (Millward, 2007).

The Uyghurs are one of the officially recognized ethnic minorities in China, and most of them live in the southern basin (Tarim Basin). The official language is Mandarin; however, other languages are spoken in Xinjiang. The Uyghur language belongs to the Karluk branch of the Turkic language family. Since ancient times, Xinjiang has been a multiethnic region and has been mentioned in Chinese records from the 206 BC to 220 AD (Millward, 2007). The Uyghurs are the main ethnic group in Xinjiang and represent 45.84% of the total population (Millward, 2007; Wyatt and Di Cosmo, 2011).

According to some historians, the Kazakh (KZK) population emerged around the 13th century. The ancestors of modern-day Kazakhs were the result of an admixture of this group with Mongol tribes from Eastern Chagatai Khanate. They speak the Kazakh language which also belongs to the Turkic language family. Till the 15th century, they were part of nomadic tribes. Kazakh is the third largest ethnic group of Xinjiang and represents 6.50% of the total Xinjiang population (Weller, 2006; Weatherford, 2012).

The article "The Heart of Silk Road “Xinjiang,” Its Genetic Portray, and Forensic Parameters Inferred From Autosomal STRs" was retracted in 2024. Reasons: lack of ethics approval or compliance; concerns about the welfare of human subjects.

Ancestors of Hui came to China from Central Asia and Islamic Persia as handicraftsmen, merchants, scholars, and soldiers. This human movement started in the seventh century and continued until the 13th century. After settling in China, they started intermingling with Han Chinese, Mongols, and Uyghurs. Ultimately, their phenotype, cultural characteristics, and language became thoroughly Chinese. Hui is the fourth largest ethnic group in Xinjiang and represents 4.51% of the total Xinjiang population (Dillon, 1999).

According to historical records, all Han Chinese can trace their origins to the Huaxia tribes which were agricultural tribes living along the Yellow River and formed during the Shang and Zhou dynasties (21st–8th centuries BC) (Cioffi-Revilla and Lai, 1995). With the rise of the Han Dynasty, all these tribes formed a common tribe/ethnic group known as the Han Chinese (Du and Vincent, 1993). Han Chinese is the world’s largest ethnic group and accounts for 18% of the worldwide population. Han is the major dominating group not only in mainland China (92%) but also in Singapore (75%). Han is the second largest ethnic group of Xinjiang and represents 40.48% of the total Xinjiang population.

DNA regions with repeat units of 2–6 bps in length are called short tandem repeats (STRs), also identified as microsatellites. STR markers are present throughout the human genome and usually have stable polymorphisms, short sequence lengths, and a dense, uniform chromosomal distribution, which makes their detection and analysis smooth using PCR and sequencing (Hammond et al., 1994; Sánchez-Diz et al., 2009). In forensic investigations such as paternity cases, rape cases, kinship analysis, and missing person analysis; STRs are considered as markers of choice because of their high polymorphism (Adnan et al., 2017; 2018b; 2018c). The Goldeneye™ 20A is a five-dye kit (Beijing PeopleSpot Inc., Beijing, China), which includes 16 combined DNA index system (CODIS) core STR loci along with Penta E, Penta D, and D6S1043 (Huang et al., 2013).

There are few studies available that focus on the characterization of autosomal STRs in the main ethnic groups of Xinjiang such as Uyghur (Yuan et al., 2016) and Kazakh (Zhang et al., 2016b). The drawbacks with previous studies are that they only focus on one or a maximum of two ethnic groups. This study focused on four main ethnic groups UGR, KZK, HUI, and HAN from Xinjiang to genotype 19 autosomal STRs using the Goldeneye 20A kit. We combined the data generated in this study with our previously published work focusing on Manchu (MCH), Mongols (MGL), Kirgiz (KGZ), and Uzbek (UZK) from Xinjiang. We then compared the genotypic data with 97 other worldwide populations.

The article "The Heart of Silk Road “Xinjiang,” Its Genetic Portray, and Forensic Parameters Inferred From Autosomal STRs" was retracted in 2024. Reasons: lack of ethics approval or compliance; concerns about the welfare of human subjects.

## 2 Materials and methods

### 2.1 Samples and DNA extraction

Blood samples were collected from 2,121 (533 Uyghur (F = 230, M = 303), 436 Kazakh (F = 204, M = 232), 593 Hui (F = 257, M = 336), and 559 Han (F = 213, M = 346) unrelated healthy individuals from the XUAR. All participants gave their informed consent either orally and with thumbprints (in case they could not write) or in writing after the study aims and procedures were carefully explained to them in their language. The study was approved by the ethical review board (dated March 20, 2019, with approval reference no. 2019-84-P) of the China Medical University, Shenyang, Liaoning Province, People’s Republic of China. All blood samples were stored at -20°C before DNA extraction. DNA was isolated from blood using the ReliaPrep™ Blood gDNA Miniprep System (Promega, Madison, WI, USA) according to the manufacturer’s instructions. The quantities of extracted DNA samples were determined using a NanoDrop spectrophotometer (Thermo Scientific, Wilmington, DE, USA), and the final concentration of DNA was diluted to 1–2 ng/μl.

### 2.2 PCR amplification

Multiplex PCR amplification of 19 autosomal STR loci (D18S51, D21S11, TH01, D3S1358, FGA, TPOX, D8S1179, vWA, CSF1PO, D16S539, D7S820, D13S317, D2S1338, D19S433, D5S818, D12S391, D6S1043, Penta D, Penta E, and the gender marker Amelogenin) was performed using the Goldeneye™ 20A kit (Beijing PeopleSpot Inc.) for all extracted DNA samples. One to 2 ng of extracted DNA was amplified according to the manufacturer’s recommended protocol. Thermal cycling was conducted in a GeneAmp PCR System 9700 thermal cycler (Applied Biosystems, Foster City, CA, USA) using the following conditions:

95°C for 5  min; 30 cycles of 94°C for 30  s, 60°C for 60  s, 70°C for 60  s; and a final extension of 60°C for 30 min.

### 2.3 Genotyping

Amplified products were prepared using the Goldeneye™ ORG 500 internal size standard (Beijing PeopleSpot Inc.) and HiDi formamide. All samples were electrophoresed using a 3,500 genetic analyzer (Applied Biosystems, Foster City, CA, USA) according to the Goldeneye™ 20A standard protocol. POP-4™ polymer (Life Technologies, Carlsbad, CA, USA) was used for capillary electrophoresis (CE). The Goldeneye™ 20A kit allelic ladder was run for each CE injection. GeneMapper™ Software version 4.0 (Life Technologies) was used for calling all alleles, which was based on the allelic ladder which followed the ISFG recommendations in this regard (Gusmão et al., 2006; Bodner et al., 2016)

### 2.4 Quality control

All extraction and quantitation batches included sterile water (sH_2_O) as negative control. Negative (sH_2_O) and positive (AmpFlSTR^®^ Control DNA 9947A) controls were employed for PCR amplification and capillary electrophoresis. All negative controls displayed an absence of amplified product while positive controls were consistent with known genotypes.

The article "The Heart of Silk Road “Xinjiang,” Its Genetic Portray, and Forensic Parameters Inferred From Autosomal STRs" was retracted in 2024. Reasons: lack of ethics approval or compliance; concerns about the welfare of human subjects.

### 2.5 Statistical analysis

The allele frequencies of STR loci, exact tests of the Hardy–Weinberg Equilibrium (HWE), and pair linkage disequilibrium tests were calculated with PowerMarker V3.25 [13]. The values for matching probability (MP), power of discrimination (PD), polymorphism information content (PIC), power of exclusion (PE) duos, typical paternity index (TPI), gene diversity (GD), and expected heterozygosity (He) were calculated by using the PowerStats software (Ver 1.2, Promega, Madison, WI, USA) [14]. Nei’s standard genetic distance between current and previously published reference populations (Law et al., 2002; Berti et al., 2005; Tie et al., 2006; Barni et al., 2007; Deng et al., 2007; Maruyama et al., 2008; Demeter et al., 2010; Stepanov et al., 2010; Zhu et al., 2010; Deng et al., 2011; Kee et al., 2011; Xing et al., 2011; Yoo et al., 2011; Chen et al., 2012; Di Cristofaro et al., 2012; Westen et al., 2012; Gaviria et al., 2013; Hedjazi et al., 2013; Nasibov et al., 2013, 2013; Park et al., 2013; Bentayebi et al., 2014; Fujii et al., 2014; Almeida et al., 2015; Gurkan et al., 2015; Parolin et al., 2015; Shafique et al., 2015; Shrivastava et al., 2015; Zhang, 2015b, 2015a; Zhang et al., 2015; Aguilar-Velázquez et al., 2016; Hossain et al., 2016; Nakamura et al., 2016; Ng et al., 2016; Park et al., 2016; Ramos-González et al., 2016; Ristow et al., 2016; Shan et al., 2016; Tokdemir et al., 2016; Vullo et al., 2016; Wang et al., 2016; Zhang et al., 2016a, 2016b; Choi et al., 2017; Guerreiro et al., 2017; Jin et al., 2017; Liu et al., 2017; Moysés et al., 2017; Ossowski et al., 2017; Perveen et al., 2017; Singh and Nandineni, 2017; Taylor et al., 2017; Wu et al., 2017; Yang et al., 2017; Adnan et al., 2018c; He et al., 2018a; Wang et al., 2018; Liu et al., 2019; Adnan et al., 2020) was computed using the Phylip 3.69 package [15]. Principal component analysis (PCA) based on allele frequency correlation and was conducted using the MVSP v3.22 software (http://www.kovcomp.com). The phylogenetic tree was constructed using MEGA X, and ancestry component dissection was explored by using STRUCTURE v.2.3.4 software (Porras-Hurtado et al., 2013). The model-based analysis employed the length of the burnin period of 100,000 and Markov Chain Monte Carlo (MCMC) step of 100,000 under the “independent allele frequencies” and “LOCPRIOR” models with the K values ranging from 2 to 10.

The article "The Heart of Silk Road “Xinjiang,” Its Genetic Portray, and Forensic Parameters Inferred From Autosomal STRs" was retracted in 2024. Reasons: lack of ethics approval or compliance; concerns about the welfare of human subjects.

## 3 Results and discussion

### 3.1 Forensic parameters

The allelic frequencies for four Xinjiang ethnic groups are summarized in Supplementary Table S1. Allelic frequencies ranged from 0.0009 (CSF1PO) to 0.5262 (TPOX) in the UGR population, ranged from 0.0011 (CSF1PO) to 0.5676 (TPOX) in KZK, ranged from 0.0008 (CSF1PO) to 0.5210 (TPOX) in HUI, and ranged from 0.0008 (D16S539) to 0.5152 (TH01) in HAN. A total of 229, 224, 229, and 232 unique alleles were observed for 19 STRs in UGR, KZK, HUI, and HAN populations, respectively. When we compared our newly studied populations on overlapping 15 STRs with our previously published data, 163, 160, 167, and 170 unique alleles were observed in UGR, KZK, HUI, and HAN, respectively, while 152, 165, 153, and 168 unique alleles were observed in the MCH, MOG, KYZ, and UZK populations, respectively. The combined powers of discrimination (CPDs) on 19 STRs were 0.999 999 999 999 999 999 999 997, 0.999 999 999 999 999 999 999 996, 0.999 999 999 999 999 999 999 993, and 0.999 999 999 999 999 999 999 983 in UGR, KZK, HUI, and HAN, respectively. The combined powers of exclusion (CPE) for 19 STRs were 0.999 999 993, 0.999 999 992, 0.999 999 988, and 0.999 999 993 in UGR, KZK, HUI, and HAN, respectively. The matching probabilities (MP) for the different populations were 2.21 × 10^−24^, 3.98 × 10^−24^, 6.05 × 10^−24^, and 1.66 × 10^−24^ in UGR, KZK, HUI, and HAN, respectively.

On combining the data for 15 STRs extracted from our previous studies for populations (MCH, MOG, KYZ, and UZK) and the current study (UGR, KZK, HUI, and HAN), CPDs were 0.999 999 999 999 999 984 833, 0.999 999 999 999 999 990 057, 0.999 999 999 999 999 996 333, 0.999 999 999 999 999 998 244, 0.999 999 999 999 999 997 679, 0.999 999 999 999 999 995 805, 0.999 999 999 999 999 993 455, and 0.999 999 999 999 999 986 23, respectively. CPEs were 0.999 999 416, 0.999 999 483, 0.999 997 932, 0.999 998 973, 0.999 998 617, 0.999 998 811, 0.999 998 151, and 0.999 998 15, respectively. CMPs for the different populations were 1/1.51 × 10^17^, 1/1.75 × 10^18^, 1/3.66 × 10^18^, 1/9.94 × 10^18^, 1/2.32 × 10^18^, 1/4.19 × 10^18^, 1/6.54 × 10^18^, and 1/1.37 × 10^17^, respectively. Penta E showed the greatest heterozygosities and PDs in all four newly studied populations. Penta E was also the most polymorphic locus in terms of alleles in the UGR (20), KZK (21), HUI (23), and HAN (21) while THO1 (6), TPOX (6), TH01 (7), and TH01 (7) were least polymorphic. Other forensic parameters such as GD, PIC, MP, PE, TPI, and Penta E loci exhibited a high level of informativeness while TPOX exhibited the least level of informativeness (Table 1). The data showed that the Goldeneye™ 20A panel can be used for forensic identification and parentage testing for the four ethnic groups in the XUAR of China.

The article "The Heart of Silk Road “Xinjiang,” Its Genetic Portray, and Forensic Parameters Inferred From Autosomal STRs" was retracted in 2024. Reasons: lack of ethics approval or compliance; concerns about the welfare of human subjects.

**TABLE 1:** Forensic parameters of the 19 autosomal STR loci in four (Uyghur, Kazakh, Hui and Han) populations residing in Xinjiang Uyghur Autonomous Region (XUAR) in China.

	CSF1PO	D12S391	D13S317	D16S539	D18S51	D19S433	D21S11	D2S1338	D3S1358	D5S818	D6S1043	D7S820	D8S1179	FGA	Penta D	PentaE	TH01	TPOX	vWA
**Uyghur**																			
No. of Alleles	10	18	7	7	18	15	18	12	8	8	16	8	10	20	12	20	6	7	9
GD	0.7375	0.8570	0.8086	0.7964	0.8656	0.8227	0.8417	0.8753	0.7456	0.7411	0.8609	0.7970	0.8281	0.8622	0.8303	0.9221	0.7779	0.6398	0.8015
PIC	0.6905	0.8402	0.7809	0.7659	0.8505	0.8006	0.8224	0.8616	0.7028	0.7002	0.8448	0.7660	0.8054	0.8461	0.8075	0.9157	0.7421	0.5905	0.7726
PM	0.1163	0.0379	0.0662	0.0741	0.0347	0.0542	0.0484	0.0307	0.1044	0.1050	0.0352	0.0704	0.0536	0.0346	0.0520	0.0137	0.0818	0.1787	0.0695
PD	0.8837	0.9621	0.9338	0.9259	0.9653	0.9458	0.9516	0.9693	0.8956	0.8950	0.9648	0.9296	0.9464	0.9654	0.9480	0.9863	0.9182	0.8213	0.9305
Hobs	0.7317	0.8612	0.7992	0.8143	0.8480	0.8180	0.8462	0.8630	0.7298	0.7148	0.8518	0.7730	0.8424	0.8424	0.8143	0.8931	0.7467	0.6454	0.7917
PE	0.4790	0.7170	0.5976	0.6258	0.6910	0.6329	0.6873	0.7207	0.4759	0.4516	0.6984	0.5499	0.6799	0.6799	0.6258	0.7813	0.5042	0.3489	0.5838
TPI	1.8636	3.6014	2.4907	2.6919	3.2901	2.7474	3.2500	3.6507	1.8507	1.7533	3.3734	2.2025	3.1726	3.1726	2.6919	4.6754	1.9741	1.4101	2.4009
**Kazakh**																			
No. of Alleles	8	15	8	7	19	13	14	14	10	8	16	9	12	16	12	21	7	6	9
GD	0.7355	0.8515	0.8196	0.8124	0.8641	0.8133	0.8138	0.8765	0.7396	0.7430	0.8661	0.7977	0.8169	0.8626	0.8293	0.9259	0.7626	0.6052	0.8106
PIC	0.6866	0.8332	0.7937	0.7839	0.8488	0.7890	0.7892	0.8627	0.6943	0.7028	0.8504	0.7660	0.7927	0.8462	0.8068	0.9198	0.7245	0.5554	0.7834
PM	0.1191	0.0399	0.0596	0.0664	0.0337	0.0597	0.0597	0.0301	0.1174	0.1059	0.0362	0.0763	0.0583	0.0354	0.0536	0.0123	0.0937	0.2111	0.0634
PD	0.8809	0.9601	0.9404	0.9336	0.9663	0.9403	0.9403	0.9699	0.8826	0.8941	0.9638	0.9237	0.9417	0.9646	0.9464	0.9877	0.9063	0.7889	0.9366
Hobs	0.7408	0.8211	0.8165	0.8165	0.8578	0.8211	0.8050	0.8647	0.7638	0.7362	0.8647	0.7936	0.7982	0.8509	0.8211	0.9151	0.7569	0.6078	0.8142
PE	0.4942	0.6388	0.6300	0.6300	0.7103	0.6388	0.6084	0.7240	0.5336	0.4865	0.7240	0.5872	0.5956	0.6967	0.6388	0.8264	0.5216	0.3003	0.6257
TPI	1.9292	2.7949	2.7250	2.7250	3.5161	2.7949	2.5647	3.6949	2.1165	1.8957	3.6949	2.4222	2.4773	3.3538	2.7949	5.8919	2.0566	1.2749	2.6914
**Hui**																			
No. of Alleles	9	14	8	7	15	15	17	14	9	9	15	11	10	20	10	23	7	7	9
GD	0.7262	0.8463	0.8133	0.7926	0.8600	0.8265	0.8154	0.8632	0.7356	0.7752	0.8744	0.7885	0.8275	0.8585	0.8214	0.9226	0.6742	0.6307	0.8038
PIC	0.6796	0.8276	0.7855	0.7608	0.8443	0.8046	0.7922	0.8474	0.6897	0.7406	0.8602	0.7573	0.8043	0.8422	0.7977	0.9164	0.6300	0.5734	0.7742
PM	0.1207	0.0425	0.0627	0.0768	0.0365	0.0545	0.0547	0.0345	0.1093	0.0890	0.0302	0.0761	0.0557	0.0365	0.0563	0.0128	0.1520	0.1942	0.0676
PD	0.8793	0.9575	0.9373	0.9232	0.9635	0.9455	0.9453	0.9655	0.8907	0.9110	0.9698	0.9239	0.9443	0.9635	0.9437	0.9872	0.8480	0.8058	0.9324
Hobs	0.7251	0.8482	0.8078	0.7892	0.8482	0.8415	0.8027	0.8398	0.7150	0.7943	0.8482	0.7774	0.8482	0.8347	0.8027	0.9174	0.6560	0.6509	0.8027
PE	0.4682	0.6914	0.6135	0.5792	0.6914	0.6782	0.6041	0.6749	0.4519	0.5884	0.6914	0.5578	0.6914	0.6650	0.6041	0.8310	0.3635	0.3565	0.6041
TPI	1.8190	3.2944	2.6009	2.3720	3.2944	3.1543	2.5342	3.1211	1.7544	2.4303	3.2944	2.2462	3.2944	3.0255	2.5342	6.0510	1.4534	1.4324	2.5342
**Han**																			
No. of Alleles	9	12	8	9	17	14	17	14	8	9	18	12	8	20	11	21	7	8	10
GD	0.7306	0.8435	0.8052	0.7874	0.8613	0.8072	0.8106	0.8624	0.7181	0.7706	0.8739	0.7759	0.8462	0.8538	0.8002	0.9218	0.6543	0.6249	0.7959
PIC	0.6862	0.8238	0.7762	0.7539	0.8453	0.7812	0.7861	0.8466	0.6677	0.7350	0.8597	0.7419	0.8263	0.8366	0.7748	0.9155	0.6085	0.5627	0.7641
PM	0.1240	0.0448	0.0680	0.0810	0.0347	0.0635	0.0588	0.0351	0.1308	0.0876	0.0313	0.0849	0.0448	0.0391	0.0655	0.0132	0.1684	0.2130	0.0724
PD	0.8760	0.9552	0.9320	0.9190	0.9653	0.9365	0.9412	0.9649	0.8692	0.9124	0.9687	0.9151	0.9552	0.9609	0.9345	0.9868	0.8316	0.7870	0.9276
Hobs	0.7585	0.8551	0.7835	0.8014	0.8479	0.8014	0.7996	0.8730	0.7138	0.7657	0.8784	0.7692	0.8533	0.8676	0.7889	0.9177	0.6708	0.6315	0.7692
PE	0.5244	0.7049	0.5689	0.6017	0.6908	0.6017	0.5984	0.7406	0.4499	0.5369	0.7515	0.5432	0.7014	0.7299	0.5786	0.8317	0.3846	0.3304	0.5432
TPI	2.0704	3.4506	2.3099	2.5180	3.2882	2.5180	2.4955	3.9366	1.7469	2.1336	4.1103	2.1667	3.4085	3.7770	2.3686	6.0761	1.5190	1.3568	2.1667

GD: gene diversity; PIC: polymorphism information content; Hobs: observed heterozygosity; PD: power of discrimination; PM: matching probability; PE: power of exclusion; TPI: typical paternity index.

The article "The Heart of Silk Road “Xinjiang,” Its Genetic Portray, and Forensic Parameters Inferred From Autosomal STRs" was retracted in 2024. Reasons: lack of ethics approval or compliance; concerns about the welfare of human subjects.

### 3.2 Hardy–Weinberg equilibrium

All of the loci were in the Hardy–Weinberg Equilibrium (HWE) in the HUI population (*p* > 0.05), while only two loci for UGR (vWA and Penta E) and one STR locus for each HAN (D13S317) and KZK (D6S1043) were out of HWE. Subsequently, when we applied sequential Bonferroni correction (Benjamini and Hochberg, 1995) to mitigate the so-called multiple comparison problem (where for a significant *p*-value of 0.05, 5% of tests are likely to be significant by chance), none of the loci in any of the four populations were found to be out of HWE (Supplementary Table S2). In our previous study (Zhan et al., 2018), none of the loci were out of HWE in the KYZ population, while one for MCH (D7S820), two for MOG (CSF1PO, D19S433), and four for UZK (D18S51, D2S1338, D7S820, and FGA) were out of HWE. However, after sequential Bonferroni correction (Benjamini and Hochberg, 1995), all loci in the four populations studied conformed to HWE.

### 3.3 Linkage equilibrium

The phenomena of linkage disequilibrium (LD) can be a result of the association between adjacent alleles co-inherited from single, ancestral chromosomes. Particularly for tightly linked genes, if a selection favors individuals with particular combinations of alleles, then it produces LD which can persist for some time. LD between two loci decays gradually in proportion to the recombination rate and time as measured in number of generations. When mutations are under positive selection, the LD surrounding the mutations is maintained because of the hitchhiking effect; thus, longer haplotypes at high frequencies can be maintained within the population. Many LD-based methods have been developed to detect positive selection. Hudson et al. (Hudson et al., 1994) proposed the first method to detect positive selection by measuring haplotype patterns. Using the extended haplotype homozygosity (EHH) test, Sabeti et al. (Sabeti et al., 2006) developed a more robust method to detect positive selection by measuring longer haplotypes at high frequencies. This method was further refined by Voight et al. (Voight et al., 2006), who standardized the EHH test using the genome-wide empirical distributions of EHH. Based on a similar rationale, Wang et al. (Wang et al., 2007) developed a new version of the LD-based method called LD decay. LD can also be caused by the rate of mutation or recombination, random genetic drift, natural selection, founder effects, nonrandom mating, recent admixture, sampling effects, and population substructure (Chakravarti, 1999). Results of exact tests for linkage equilibrium (LE) displayed that *p*-values of 116 pairwise combinations of STR loci (UGR 32, KZK 31, HUI 32, and HAN 21) were lower than 0.05 and thus showing LD (Supplementary Table S3). Subsequently, when we applied sequential Bonferroni correction (Benjamini and Hochberg, 1995), only 17 pairs were out of LE. These pairs were D6S1043/D2S1338, D2S1338/D5S818, D18S51/D21S11, D12S391/TPOX, TPOX/Penta D, and D6S1043/D5S818 in the UGR population; D7S820/FGA, D18S51/D8S1179, D7S820/Penta E, CSF1PO/D3S1358, and D6S1043/D8S1179 in the KZK population; D2S1338/D5S818, TH01/D18S51, D12S391/FGA, and D13S317/TH01 in the HUI population; and CSF1PO/D3S1358 and FGA/CSF1PO in the HAN population. We tested 171 pairwise LE tests in each population, and a maximum of six was out of LE in each population. The product rule is used to estimate the random chance of detecting a given STR profile within a population. This is done by multiplying the frequencies of each of the genotypes (combination of alleles) found at all loci in the STR profile (Butler and Butler, 2010). Presentation of the “product rule” for calculating the RMP across multiple STRs can be seen in the HAN population (only two pairs were out of LE) while in the other three (UGR, KZK, and HUI) populations it was unlikely to produce significant errors. The HAN population is not an endogamous population while the other three are endogamous populations. There is no trend of external mating in Xinjiang Muslim populations. The same results were observed in our previous study for the Kyrgyz and Uzbek populations.

The article "The Heart of Silk Road “Xinjiang,” Its Genetic Portray, and Forensic Parameters Inferred From Autosomal STRs" was retracted in 2024. Reasons: lack of ethics approval or compliance; concerns about the welfare of human subjects.

### 3.4 Ancestry content analysis with structure

STRUCTURE analysis (which uses model-based clustering algorithm) was done for four populations (Xinjiang Han, Uyghur, Kazakh, and Xinjiang Hui) and publicly available data for seven populations (Mongol, Kyrgyz, Uzbek, Manchu, Liaoning Han, Tibetan, and Jilin Korean). The data were used to explore ancestry content and genetic landscapes of Xinjiang populations. The number of inferred clusters (K) varied from 2 to 10 with 10 repetitions of each K value and a total of 10,000 burnins and 10,000 Markov chain Monte Carlo (MCMC) simulations for each repetition. We observed that the best optimal number of ancestral populations was five (K = 5). Uyghur and Kazakh populations shared most of their genetic components with other Turkic-speaking populations such as Uzbek and Kyrgyz (yellow) while they shared a few genetic components with Tibetan (blue) and Han, Hui, Munch, and Korean populations (pink) (Figure 1). The pink component was a common component that was present in all populations studied. Moreover, two genetic clusters were observed. One cluster mainly contained populations that are descendants of ancient Altai-speaking populations, and the second cluster contained mainly East Asian populations. Uyghur and Kazakh populations appeared to be genetically closer to Altai-speaking populations while Han and Hui populations were closer to East Asian groups. Results of K2-10 are shown in Supplementary Figure S1. PCA on raw genotype data of 11 populations showed 1.39% of variations, while in the second component, 0.95% of variations were observed. We observed two main clusters on these two (1&2) components: the first cluster contains Kyrgyz, Kazakh, and Mongol populations, while the second cluster contains Uzbek, Uyghur, Manchu, Hui, Tibetan, Korean, and Han populations. On PC1 and PC3 (0.87%), a total of 2.26% of variations were observed. Here we observed three clusters. The first cluster contained Kyrgyz, Kazakh, and Mongol populations. The second cluster had Uzbek, Uygur, and Tibetan populations. In the third cluster, typical East Asian populations (Han, Hui, Manchu, and Korean) were grouped together.

The article "The Heart of Silk Road “Xinjiang,” Its Genetic Portray, and Forensic Parameters Inferred From Autosomal STRs" was retracted in 2024. Reasons: lack of ethics approval or compliance; concerns about the welfare of human subjects.

**FIGURE 1:** Genetic structure and population relationship between Xinjiang Han, Uyghur, Kazakh, Hui, Manchu, Kyrgyz, Uzbek, Mongol, and other Chinese populations.

PC2 (0.95%) and PC3 (0.87%) resulted in three clusters. In the first cluster, only the Tibetan population was grouped while in the second and third clusters all Altai-speaking populations and typical East Asian populations were present, respectively. PC1 and PC4 (0.84%) also gave us interesting results. Here, two clusters were formed. In the first cluster, the Tibetan population along with typical East Asian populations was grouped while in the second cluster all Altai-speaking populations were present. Results of PCA (Figure 2) were in support with STRUCTURE analysis. These results were also consistent with linguistic affinity and also whole-genome sequencing and high-density genotyping data (Xu et al., 2008; Xu and Jin, 2008; Bai et al., 2018).

**FIGURE 2:** Principal component analysis (PCA) revealed the genetic relationship on the basis of the first four components between Xinjiang Han, Uyghur, Kazakh, Hui, Manchu, Kyrgyz, Uzbek, Mongol, and other Chinese populations.

### 3.5 Xinjiang and worldwide population comparison

We have compared the data of four populations with previously published populations from Xinjiang of northwest China and worldwide regions using AMOVA, employing available data for 15 STR loci. Genetic distances between the HAN population and 12 other populations from Xinjiang (Xinjiang Uyghur, Xinjiang Hui, Xinjiang Kazakh, Xinjiang Kyrgyz, Xinjiang Manchu, Xinjiang Uzbek, Xinjiang Mongols, Uygur-Xinjiang-1, Kazakh-Xinjiang-1, Kumul-Uyghur-Xinjiang-3, Uyghur-Xinjiang-2, Kazakh-Xinjiang-2) based on Nei’s standard formula are listed in Supplementary Table S4A. These Nei’s standard genetic distance values were used to build a neighbor-joining tree (N-J tree) between Xinjiang Han and 12 other populations (Figure 3A). The Hui population (0.0046) from Xinjiang showed the closest genetic distance with HAN followed by the Mongol population (0.0244) from Xinjiang, while the Kazakh-1 population (1.1693) showed the greatest genetic distance which is followed by the Kyrgyz population (0.4547) from Xinjiang. The first three components (extracting 91.13% genetic variations) of PCA based on allelic frequencies of 15 STRs showed that Altai-speaking populations were closely linked **(** Figure 3B **)**. A heat map (Figure 3C) using the genetic distances showed two clusters. In the first cluster, Manchu, Kyrgyz, Uzbek, and Kazakh-1 were grouped together while the second cluster contained other nine populations. According to Zhang et al. (Zhang et al., 2016a), Uyghurs are genetically closer to the central Asian population and Mongolian populations from East Asia. Jin et al. (Jin et al., 2017) found that these Turkic language-speaking groups placed themselves in the middle of European and East Asian populations. Feng et al. (Feng et al., 2017) used genome-wide human SNP array and found that the Uyghur population from XUAR have four major ancestral components, which were the result of two earlier admixed groups: one of them was from the West containing European (25%–37%) and West South Asian ancestries (12–20%), while the second one was from the East, with Siberian (15%–17%) and East Asian (29%–47%) ancestries. Results of MultiWaver showed us a two-wave admixture. The earliest wave was ∼3,750  years ago (ya), and a recent wave ∼750 ya. According to Seidualy et al. (Seidualy et al., 2020), the Kazakh population has a mixed ancestry containing East Asian (32.8%), European (30.8%), North Asians (28.9%), and South Asians (6%). Wen et al. (Wen et al., 2021) found that the Northwest Chinese Kyrgyz showed a high percentage of Y haplogroup R1a1a1b2a2a-Z2125, which is related to Bronze Age Siberians, while the second dominant haplogroup was C2b1a3a1-F3796, related to Medieval Niru’un Mongols, such as the Uissun tribe from Kazakhs. Again, Wen et al. (Wen et al., 2020) found that the Kazakh population from China showed the highest frequency (80%) of haplogroup C2b1a3a1-F3796 (previous C3*-Star Cluster) which is predominantly found in Mongolian descendent populations. Wang et al. (Wang et al., 2019) found that the Hui population has about 70% in total of the paternal ancestry which could be traced back to East Asia and the left 30% to various regions in West Eurasia. Zhao et al. (Zhao et al., 2020) investigated that Mongolian and Kazakh groups derived 6%–40% of their ancestry from West Eurasia while 42%–64% of their ancestry was from East Asia. He et al. (He et al., 2018b) reported that the Uygur population has 36.30% of European-related ancestry while Hui only have 3.66% of it. Liu et al. (Liu et al., 2018) reported that the Tibetan population and Hui population have a genetic affinity with East Asian populations, while the Uygur population showed a similar genetic makeup with South Asian populations.

The article "The Heart of Silk Road “Xinjiang,” Its Genetic Portray, and Forensic Parameters Inferred From Autosomal STRs" was retracted in 2024. Reasons: lack of ethics approval or compliance; concerns about the welfare of human subjects.

**FIGURE 3:** **(A)** A Neighbor-joining tree explaining the phylogenetic relationship between Xinjiang populations. **(B)** A heat map of pairwise Nei’s genetic distance values between Xinjiang populations. **(C)** Principal component analysis (PCA) based on Nei’s genetic distance revealed by the first two components between Xinjiang populations.

Genetic distances among the HAN population and 104 worldwide populations were calculated using Nei’s standard formula and summarized in Supplementary Table S3D. Among worldwide populations, Asians living in Australia (0.0123) showed the closest association with the HAN population followed by the Chamorro population (0.0574); on the other hand, the Haitian population (0.2322) showed a distant association followed by the amaXhosa population (0.2251) from South Africa. These Nei’s genetic distance values were used to build a neighbor-joining tree (N-J tree) between Xinjiang Han and 104 worldwide populations (Figure 4). The first 10 components of PCA (PC1 = 25.06%, PC2 = 14.70%, PC3 = 9.80%, PC4 = 6.55%, PC5 = 6.02%, PC6 = 5.40%, PC7 = 4.19%, PC8 = 3.07%, PC9 = 2.39% and PC10 = 2.08%) extracted 79.31% of genetic variations (Figure 5). A heat map of the genetic distance matrix was also generated among 105 worldwide populations (Figure 6). Populations from Xinjiang showed their affinity with Central Asian, South West Asian, West Asian, and East European populations. An interactivity test between these 105 worldwide populations showed that the results were consistent with the PCA and Nei’s formula results described above (Figure 7). Comparisons between only Chinese ethnic groups (Supplementary Figures 2A–C) and Asian ethnic groups (Supplementary Figure 3–C) are discussed in Supplementary Text S1.

**FIGURE 4:** A Neighbor-joining tree explaining the phylogenetic relationship between Xinjiang Han population and 104 other reference populations from worldwide.

**FIGURE 5:** A heat map of pairwise Nei’s genetic distance values between Xinjiang Han population and 104 other reference populations worldwide.

**FIGURE 6:** Principal component analysis (PCA) based on Nei’s genetic distance revealed by the first two components between the Xinjiang Han population and 104 other reference populations from worldwide.

**FIGURE 7:** Interactivity test between the Xinjiang Han population and 104 other reference populations from worldwide.

## 4 Conclusion

In the current study, we genotyped 20 autosomal STR loci in the Han, Uyghur, Kazakh, and Hui ethnic groups of Xinjiang and calculated the forensic parameters. The Goldeneye^®^ 20A panel appeared suitable for forensic investigations such as personal identification and paternity testing and had a high power of discrimination. The STR loci included in the kit showed no significant departures from HWE and minimal departure from LE for a very small number of pairwise combinations of loci. Genetic characterization showed that the Uyghur and Kazakh ethnic groups were closely related to other Turkic-speaking groups while the Han and Hui populations showed their associations with other Sinitic language-speaking populations. Interestingly, the Kazakh population showed an affinity with the Mongols which suggested an ancient divergence between Kazakh and Mongols when Mongols originally migrated to present-day Xinjiang (Adnan et al., 2018a; Zhan et al., 2018; He et al., 2019).

The article "The Heart of Silk Road “Xinjiang,” Its Genetic Portray, and Forensic Parameters Inferred From Autosomal STRs" was retracted in 2024. Reasons: lack of ethics approval or compliance; concerns about the welfare of human subjects.

## Data Availability

The original contributions presented in the study are included in the article/Supplementary Material; further inquiries can be directed to the corresponding authors.
